# Effectiveness of Inexpensive Cloth Facemasks and Their Amendments to Reduce Ambient Particulate Exposures: A Case of Kathmandu, Nepal

**DOI:** 10.1155/2023/5144345

**Published:** 2023-01-31

**Authors:** Prasidha R. Neupane, Iswor Bajracharya, Sunil B. Khatry

**Affiliations:** ^1^Khwopa College (Tribhuvan University), Bhaktapur, Nepal; ^2^Nepal Academy of Science and Technology (NAST), Lalitpur, Nepal; ^3^Nepal Environmental Scientific Services (P) Ltd (NESS), Baneshwor, Nepal

## Abstract

Inexpensive cloth masks are widely used to reduce particulate exposures, but their use became ubiquitous after the outbreak of COVID-19. A custom experimental setup (semiactive at 5.1 m/s airflow rate) was fabricated to examine the efficiency of different types of commercial facemasks collected randomly from street vendors. The sample (*N* = 27) including (*n* = 16) cloth masks (CMs), (*n* = 7) surgical masks (SMs), and (*n* = 4) N95 filtering facepiece respirators (FFRs), of which SMs and N95 FFRs taken as a standard for efficiency comparison were all tested against ambient aerosols (PM_2.5_ and PM_10_ *μ*g/m^3^). The prototype cloth masks (PTCMs) (*N* = 5) design was tailored, and their performance was assessed and compared with that of standard commercial masks. The filtering efficiency tested against ambient coarse particulates (PM_10_) ranged from (5% to 34%) for CMs with an average of 16%, (37% to 46%) for SMs with an average of 42%, (59% to 72%) for PTCMs with an average of 65%, and (70% to 75%) for N95 FFRs with an average of 71%, whereas against fine particulates (PM_2.5_), efficacy ranged from (4% to 29%) for CMs with an average of 13%, (34% to 44%) for SMs with an average of 39%, (53% to 68%) for PTCMs with an average of 60%, and (68% to 73%) for N95 FFRs with an average of 70%, respectively. The efficiency followed the order N95 FFRs > PTCMs > SMs > CMs showing poor exposure reduction potential in CMs and high exposure reduction potential in N95 FFRs and PTCMs. Amendment in existing CMs using eco-friendly cotton fabric with better facial adherence can protect human health from exposure to fine particulates <2.5 *μ*m and can reduce the risk of micro-plastic pollution caused by polypropylene (PP) facemasks.

## 1. Introduction

The bowl-shaped topographic structure in Kathmandu Valley is surrounded by mountains that are impediments to wind movement that retains particulates in ambient air [1, 2], which is a key indicator of air pollution [3]. Traffic-related particulate matter (PM) is considered a major contributor to overall ambient air pollution in Nepal [4, 5], causing adverse impacts on the health of commuters and pedestrians due to their proximity to vehicular emissions [6, 7] and also being responsible for an alteration of climate and visibility [8]. Particulate matter (PM) exposure is associated with respiratory and cardiovascular health effects [9–11] along with premature mortality [12, 13], which reflects global health concerns [14, 15]. In Nepal, 24,000 premature annual deaths are expected to happen by 2030 due to ambient air pollution [16].

Long-term policies such as shifting to clean energy and short-term policies such as population-level interventions such as the use of respiratory protective devices (RPDs) might be the two effective approaches to reduce particulate exposures and other harmful airborne contaminants [5, 17, 18]. Application of RPDs has played a significant role as a first-hand transmission controlling agent throughout history such as in the cases of acute respiratory syndrome coronavirus-1 (SARS-CoV-1) in 2003 [19], influenza H191 in 2009 [20], avian H5N1 in 2003 [21], Ebola virus in 2014 [22], and Middle East respiratory syndrome coronavirus (MERS-CoV) in 2012 [23], respectively. The surge in the use of facemasks took place after the outbreak of severe acute respiratory syndrome coronavirus-2 (SARS-CoV-2) also known as COVID-19 from China [24, 25] and was recognized as a pandemic by the WHO on 11 March, 2020 [26, 27]. Facemasks were the only precaution taken during the COVID-19 pandemic [28–30] due to the limited supply of vaccines to meet global demand [31], resulting in global shortages of commercial facemasks and personal protective equipment (PPE) for healthcare workers (HCWs) [32–34].

Anecdotal evidence showed that during the Manchurian epidemic, handmade masks of cotton gauze became useful for military barracks and healthcare workers when quality commercial masks were inaccessible [35, 36]. Simple, locally made, washable cloth masks (CMs) are suggested for use as an alternative when deprived of commercial masks [37, 38]. The researchers advocated for the public's use of CMs as a complementary countermeasure to the current COVID-19 pandemic [39–41] and they are being embraced worldwide [42]. Although limited scientific data existing on the efficacy of CMs [43], people are using them because they are reusable and cheaper than surgical masks (SMs) and N95 filtering facepiece respirators (FFRs) [44, 45]. The efficacy of commercial facemasks certified to local or international standards such as N95 FFRs and SMs are considered superior compared to that of CMs [28, 46, 47], but in some cases, their performance may not meet the exposure reduction potential that is marketed commercially [48]. The efficiency of facemasks against aerosols (viral or pollution particles) varies due to the different sizes, shapes, and properties of the particles [17]. The efficiency of facemasks is also affected by factors such as the charge of the aerosol, types of mask material, pollutant concentration, airflow rate, size and shape of the human face, facial hair, and way of wearing [48–50].

Very few studies have been done in Nepal regarding evaluating the efficacy of facemasks. The study carried out by Shakya et al. [43] evaluated three CMs and one SM, and Neupane et al. [5] evaluated twenty CMs and seven SMs, which resulted in the efficacy of CMs being inferior. However, their study lacks providing insights regarding the improvement in CMs whose performance can be equivalent to that of standard commercial masks. This study gives an overview of the efficacy of CMs and the efficacy of their amended version known as prototype cloth masks (PTCMs) in this study as well as makes a comparison with the efficacy of SMs and N95 FFRs, which are taken as standards in this study. The motivation for developing PTCMs in this study is to encourage people to use eco-friendly cotton facemasks with a better facial fit that have similar exposure reduction potential as polymer-based standard commercial facemasks that are a source of microplastic pollution.

## 2. Materials and Methods

This experiment was conducted in 2020 from February to March and August to November, consecutively, at the open ground of North Valley School, Kathmandu. As humans are naturally exposed to the ambient atmosphere, the experiment was conducted by extracting natural ambient aerosols in sealed setups (Figure 1).

This experimental setup was fabricated using a normal plyboard, polyvinyl chloride (PVC) pipe, computer fan, revolutions per minute (RPM) controller, and a 12 V (volt) direct current (DC) charger. Ambient fine particulates (PM_2.5_) and coarse particulates (PM_10_) in real-time concentration (*μ*g/m^3^) were extracted at 5.1 m/s (stagnant air flow rate) and tested with two calibrated portable hand-held detectors (BR-Smart series model with an inbuilt light scattering measurement method, resolution: 1 *μ*g/m^3^, and accuracy: ±10) simultaneously between filtrate air (with facemask) and nonfiltrate air (without a facemask).

### 2.1. Sample Size

Twenty-seven nasopharyngeal masks (*N* = 27), which includes CMs (*n* = 16), SMs (*n* = 7), and N95 FFRs (*n* = 4), were randomly collected from street vendors. The SMs and N95 FFRs were used as standards in this study for efficiency comparison.

### 2.2. Efficiency Estimation Equation

The filtering efficiency of facemasks was calculated using (1) referred to in the previously published studies [48, 51].

(1) $$\begin{array}{c} \text{effectiveness}=\frac{\text{no mask}-\text{with mask}}{\text{no mask}}\times 100\%, \end{array}$$

where “no mask” is the particles measured without wearing a mask, and “with mask” is the particles measured while wearing a mask on a human mannequin head.

### 2.3. Stitching of Prototype Cloth Masks (PTCMs)

Five different designs of cloth masks were conceptualized and stitched with the collaboration of a local garment factory in Kathmandu, Nepal (Table 1).

The PTCMs were stitched using a few varieties of cotton fabrics in all five designs with the addition of a few accessories such as adjustable ear straps and nose pin for better facial adherence, pockets for inserting filters made of either polypropylene (PP) fabric or tissue paper as per the user's convenience.

## 3. Results

The filtering efficacy of tested surgical masks (SMs) against PM_10_ ranged from 37% to 46%, with the lowest efficacy found on SM4 (37%), and the highest efficacy found on SM6 (46%) (Table 2). The highest filtering efficiency in SM6 was found to reduce PM_10_ concentration from 34.7 ± 2.37 *μ*g/m^3^ to 18.9 ± 4.32 *μ*g/m^3^ with a total inward leakage (TIL) of 54%. The average filtering efficacy of SMs against ambient PM_10_ was found to be 42%.

The filtering efficacy of tested SMs against PM_2.5_ ranged from 34% to 44%, with the lowest efficacy found on SM4 (34%), and the highest efficacy found on SM6 (44%) (Table 3). The highest filtering efficiency in SM6 was found to reduce PM_2.5_ concentration from 20.6 ± 1.31 *μ*g/m^3^ to 11.5 ± 3.72 *μ*g/m^3^ with a total inward leakage (TIL) of 56%. The average filtering efficacy of SMs against ambient PM_2.5_ was found to be 39%.

The filtering efficacy of tested CMs against PM_10_ ranged from 5% to 34%, with the lowest efficacy found on CM13 (5%) and the highest efficacy found on CM14 (34%) (Table 4). The highest filtering efficiency in CM 14 was found to reduce PM_10_ concentration from 61.48 ± 5.79 *μ*g/m^3^ to 40.3 ± 8.47 *μ*g/m^3^ with a total inward leakage (TIL) of 66%. The average filtering efficacy of CMs against ambient PM_10_ was found to be 16%.

The filtering efficacy of tested cloth masks against PM_2.5_ ranged from 4% to 29% with the lowest efficacy found on CM 13 (4%) and the highest efficacy found on CM 14 (29%) (Table 5). The highest filtering efficiency in CM 14 was found to reduce PM_2.5_ concentration from 49.64 ± 5.75 *μ*g/m^3^ to 35.15 ± 5.58 *μ*g/m^3^ with a total inward leakage (TIL) of 71%. The average filtering efficacy of CMs against ambient PM_2.5_ was found to be 13%.

The filtering efficiency of N95 filtering facepiece respirators (FFRs) against PM_10_ ranged from 70% to 75%, with the lowest filtering efficiency found on N95 (i), N95 (ii), and NIOSH respirator (70%) and the highest filtering efficiency found on N95 (iii) (75%) at an airflow rate of 5.1 m/s (Table 6). The highest filtering efficiency in the N95 (iii) mask was found to reduce PM_10_ concentration from 131.7 ± 24.12 *μ*g/m^3^ to 33.31 ± 26.74 *μ*g/m^3^ with a total inward leakage (TIL) of only 25%. The average filtering efficacy of N95 FFRs against ambient PM_10_ was found to be 71%.

The filtering efficiency of N95 FFRs against PM_2.5_ ranged from 68% to 73%, with the lowest filtering efficiency found on N95 (ii) (68%), and the highest filtering efficiency found on N95 (iii) (73%) (Table 7). The highest filtering efficiency in the N95 (iii) mask was found to reduce PM_2.5_ concentration from 138.1 ± 22 *μ*g/m^3^ to 36.75 ± 20.43 *μ*g/m^3^ with a total inward leakage (TIL) of 27%. The average filtering efficacy of N95 FFRs against ambient PM_2.5_ was found to be 70%.

The filtering efficacy of prototype cloth masks (PTCMs) against PM_10_ ranged from 59% to 72%, with the lowest efficacy found on PTCM4 (59%) and the highest efficacy found on PTCM1 (72%) (Table 8). The highest filtering efficiency in PTCM1 was found to reduce the 95% CL level of PM_10_ concentration from 49.98 ± 2.83 *μ*g/m^3^ to 13.82 ± 3.35 *μ*g/m^3^ with a total inward leakage (TIL) of 28%. The average filtering efficacy of PTCMs against ambient PM_10_ was found to be 65%.

The filtering efficacy of prototype cloth masks (PTCMs) against PM_2.5_ ranged from 53% to 68%, with the lowest efficacy found on PTCM4 (53%), and the highest efficacy found on PTCM1 (68%) (Table 9). The highest filtering efficiency in PTCM1 was found to reduce the 95% CL level of PM_2.5_ concentration from 41.64 ± 2.1 *μ*g/m^3^ to 13.49 ± 3.34 *μ*g/m^3^ with a total inward leakage (TIL) of 68%. The average filtering efficacy of PTCMs against ambient PM_2.5_ was found to be 60%.

The average filtering efficacy of SMs, CMs, PTCMs, and N95 FFRs nasopharyngeal masks against ambient PM_10_ were found at 42%, 16%, 65%, and 71%, whereas against ambient PM_2.5_ average efficiency of SMs, CMs, PTCMs, and N95 FFRs were found at 39%, 13%, 60%, and 70%, respectively (Figure 2).

The more was efficiency found the lesser the total inward leakage (TIL) for particulate filtration at the stated airflow rate. The efficiency followed the order N95 FFRs > PTCMs > SMs > CMs showing poor exposure reduction potential in CMs and high exposure reduction potential in N95 FFRs and PTCMs.

### 3.1. Statistical Analysis

Karl Pearson's correlation (*r*) analysis between variables showed a significant positive correlation (*r* = 0.92, *p* < 0.05) between number of mask layers and efficiency (PM_10_) and correlation (*r* = 0.94, *p* < 0.05) between number of mask layers and efficiency (PM_2.5_), respectively (Table 10).

One-way analysis of variance (ANOVA) test showed that the efficiency of all face masks against PM_10_ and PM_2.5_ are found to be significantly different from each other (*p* < 0.01), which rejected the null hypothesis of this study.

## 4. Discussion

The efficacy of nasopharyngeal masks was estimated using different methods and techniques in previous studies, which contradict each other because different studies used different methods and experimental approaches whose findings varied from study to study although studied for the same subject [7]. The applied nasopharyngeal masks were found slightly better in efficiency for ambient PM_10_ aerosols than PM_2.5_ due to the size and shapes of the aerosols [17].

Poor facial fit increases the particulate penetration level known as total inward leakage (TIL) [48, 52] at different breathing frequencies [50] and particle penetration level decreases with increasing particle size [53, 54]. The TIL values were found to be low in SMs and N95 FFRs compared to CMs in our study and previous studies [55, 56]. It is found that the efficacy of CMs widely varied from each other due to large pore size in CMs allowing particulates to pass easily, however, it performed well for larger particles >300 nm [42] and is believed to impede droplets and aerosols transmission [57]. The filtering efficiency of CMs ranging from 5% to 34% in our study has a close agreement with the efficacy range of 5% to 25% [58], 7% to 66% [48], 5% to 57% [43], and 34% to 66% [59], respectively. The variation in efficacy can be attributed to the factors such as facial adherence, fabric material, airflow rate [48–50, 60], and the sizes, shapes, and properties of aerosols [17].

The efficacy of SMs was found better than that of CMs because it has similar surface characteristics as N95 FFRs embedded with a complex network of polypropylene (PP) nanofibers forming web-like structures interconnected with each other [5] and is triboelectrically charged to enhance the filtering efficacy by 6% to more than 10% [58]. However, its performance can decline in high airflow rate conditions due to its poor facial adherence (a gap between the nasal bone and face) [48, 52], but can be improved if modified with a better facial fit [61].

N95 FFRs, characterized by a complex network of multiple layers of nanofibers forming a web-like structure, melt-blown filters, and better facial adherence over the face [37, 47, 62] stand superior in reducing particulate exposures in our studies as well as in the previous study [46, 63, 64] that showed it is more capable of preventing nanoparticles from penetrating through its fabrics [65]. The efficacy of N95 FFRs for coarse particulate matter ranging from 70% to 75% in our study has a close agreement with the efficacy range of 3.5% to 68.1% [46], whereas for fine particulate matter ranging from 68% to 73% in our study has a close agreement with the efficacy range of 14% to 96% [6].

The filtering efficacy of PTCMs against fine particulates ranging from 53% to 68% in our study has a close agreement with the filtering efficacy ranged from 20% to 60% against fine NaCl particles [28]. The average filtering efficiency of PTCMs against fine particulates 60% in our study, which is in close agreement with the 45% average efficacy of layered fabrics [66]. The stacking of different fabric layers in PTCMs played a significant role in reducing incoming particulates through fabrics in our study, as suggested by the study, of Drewnick et al., Zangmeister et al., and O'Kelly et al. [66–68]. The better filtering efficiency shown by N95 FFRs and SMs against various sizes of particulate matter [28, 46, 69] are sources of plastic pollution [70–72] because they are polymer products [73, 74]. Such PP facemasks harm the environment, human health, and aquatic life and can jeopardize global food safety [75–77]. N95 FFRs are costly and cannot be reused multiple times. The PTCMs in this study are made of cotton fabrics and are purely eco-friendly.

These modified reusable CMs featured adjustable ear loops, pockets for installing replaceable filters, a nose pin for better facial fit, and some fabric layers for better filtration of particulate exposures, resulting in an efficacy almost equivalent to N95 FFRs. Such designs can be embraced by people when commercial facemasks are shortened or not available [59, 66].

## 5. Conclusions

The filtering performance of CMs was found to have poor exposure reduction potential and is marginally beneficial to human health compared to SMs and N95 FFRs. However, few amendments in inexpensive cloth mask materials and design that fits replaceable filters inside, whether PP filter or tissue paper as per that user's convenience, with the installation of a few accessories like a nose pin and adjustable ear straps for better adherence to the human face resulted in efficacy almost equivalent to standard N95 FFRs. The findings suggest that PTCMs can be potential alternatives to expensive standard masks and can play a pivotal role in reducing harmful ambient particulate exposures. The findings of this study can be helpful for the government to formulate policies and guidelines for better use of eco-friendly facemasks as well as it can also help the public regarding the proper selection of facemasks. Eco-friendly facemasks with better efficacy should be brought into mass production to replace plastic-based facemasks to protect both the environment and human health.

### 5.1. Limitations

In the semiactive measurement experiment setup (Figure 1), the air inlet was maintained at 5.1 m/s, but an air outlet was not made, as well as the setups were not fully sealed, on the other hand the facemask sample testing zone was such that it stretched the fabric in some extent, which these all conditions favors the leakage of incoming PM particulates from both the fabric and the experimental setups. The leakage source other than from fabric which acted as a confounding factor in this experiment was not measured. Because of these conditions, the efficiency values were underestimated even for standard N95. More detailed studies are required to justify confounding factors that influence the efficacy of facemasks.

## Figures and Tables

**Figure 1:** Schematic diagram of semiactive custom experimental setup for measuring the efficacy of nasopharyngeal masks.

**Figure 2:** Average filtering efficiency of facemasks.

**Table 1:** Accessories and materials for prototype cloth masks (PTCMs).

S. N.	PTCMs	Fabric types	Material components	Total layers	Price, NRs
1	P1	Cotton	Filter, stretchable ear loop, nose pin	4	50
2	P2	Cotton	Filter, adjustable ear loop	4	50
3	P3	Sinker	Filter, adjustable ear loop, nose pin,	4	50
4	P4	Sinker	Filter, net, nose pin, adjustable ear loop	4	50
5	P5	Sinker	Foam, filter, nose pin, adjustable ear loop	4	50

**Table 2:** Filtering efficiency of SMs against PM_10_.

S. N.	Surgical masks (SMs)	Without filtration (*μ*g/m^3^) mean ± S.D	With filtration (*μ*g/m^3^) mean ± S.D	TIL (%)	Efficiency (%)
1	SM 1	30 ± 14.59	17.5 ± 10.5	58	42
2	SM 2	32 ± 10.4	17.5 ± 4.67	55	45
3	SM 3	34.3 ± 2.44	20.1 ± 2.67	59	41
4	SM 4	36 ± 4.75	22.7 ± 6.22	63	37
5	SM 5	32.9 ± 2.02	18.5 ± 3.04	56	44
6	SM 6	34.7 ± 2.37	18.9 ± 4.32	54	46
7	SM 7	33.9 ± 14.41	21.1 ± 14.3	62	38

**Table 3:** Filtering efficiency of SMs against PM_2.5_.

S. N.	Surgical masks (SMs)	Without filtration (*μ*g/m^3^) mean ± S.D	With filtration (*μ*g/m^3^) mean ± S.D	TIL (%)	Efficiency (%)
1.	SM 1	20 ± 13.55	12.4 ± 10.32	62	38
2.	SM 2	28 ± 7.36	16.2 ± 4.32	58	42
3.	SM 3	26 ± 1.99	16 ± 2.52	62	38
4.	SM 4	25.8 ± 3.01	17.1 ± 6.06	66	34
5.	SM 5	21.6 ± 1.23	12.5 ± 2.76	58	42
6.	SM 6	20.6 ± 1.31	11.5 ± 3.72	56	44
7.	SM 7	24.3 ± 14.23	15.6 ± 12.9	63	37

**Table 4:** Filtering efficiency of CMs against PM_10_.

S. N.	Cloth masks (CMs)	Without filtration (*μ*g/m^3^) mean ± S.D	With filtration (*μ*g/m^3^) mean ± S.D	TIL (%)	Efficiency (%)
1.	CM 1	82.23 ± 7.34	63.62 ± 2.5	77	23
2.	CM 2	70.02 ± 7.32	49.71 ± 2.54	71	29
3.	CM 3	91.56 ± 7.28	61.23 ± 3.36	67	33
4.	CM 4	82.13 ± 19.59	62.34 ± 5.57	76	24
5.	CM 5	64.73 ± 8.85	56.82 ± 5.92	88	12
6.	CM 6	61.82 ± 2.16	53.38 ± 1.7	86	14
7.	CM 7	64.62 ± 1.9	59.63 ± 1.85	92	8
8.	CM 8	56.27 ± 2.35	50.59 ± 3.8	90	10
9.	CM 9	65.13 ± 2.51	59.7 ± 1.62	92	8
10.	CM 10	66.7 ± 3.48	61.79 ± 1.96	93	7
11.	CM 11	40.9 ± 22.87	33.97 ± 18.35	83	17
12.	CM 12	17.69 ± 3.38	16.19 ± 9.59	92	8
13.	CM 13	99.83 ± 28.56	94.5 ± 26.14	95	5
14.	CM 14	61.48 ± 5.79	40.3 ± 8.47	66	34
15.	CM 15	109 ± 138.37	95.53 ± 156.66	88	12
16.	CM 16	50.75 ± 15.16	44.66 ± 15.57	88	12

**Table 5:** Filtering efficiency of CMs against PM_2.5_.

S. N.	Cloth masks (CMs)	Without filtration (*μ*g/m^3^) mean ± S.D	With filtration (*μ*g/m^3^) mean ± S.D	TIL (%)	Efficiency (%)
1.	CM 1	87.98 ± 6.84	73.15 ± 4	83	17
2.	CM 2	78.36 ± 8.17	61.41 ± 1.99	78	22
3.	CM 3	98.2 ± 6.65	71.26 ± 4.55	73	27
4.	CM 4	88.33 ± 18.69	72.08 ± 8.68	82	18
5.	CM 5	74.07 ± 11.42	67.98 ± 7.47	92	8
6.	CM 6	49.58 ± 1.6	43.93 ± 1.27	89	11
7.	CM 7	51.64 ± 1.56	48.15 ± 1.38	93	7
8.	CM 8	68.69 ± 3.05	62.87 ± 2.71	92	8
9.	CM 9	52.16 ± 2.24	48.28 ± 1.14	93	7
10.	CM 10	53.62 ± 4.3	49.64 ± 1.46	93	7
11.	CM 11	36.38 ± 19.92	30.56 ± 14.96	84	16
12.	CM 12	15.95 ± 2.6	14.75 ± 8.63	92	8
13.	CM 13	93.32 ± 26.34	89.52 ± 24.8	96	4
14.	CM 14	49.64 ± 5.75	35.15 ± 5.58	71	29
15.	CM 15	124.5 ± 115.76	111.6 ± 135.25	90	10
16.	CM 16	42.15 ± 10.31	37.8 ± 11.19	90	10

**Table 6:** Filtering efficiency of N95 FFRs against PM_10_.

S. N.	N95 FFRs	Without filtration (*μ*g/m^3^)	With filtration (*μ*g/m^3^)	TIL (%)	Efficiency (%)
1.	N95 (i)	60.32 ± 4.46	17.97 ± 3.27	30	70
2.	N95 (ii)	5.34 ± 1.67	1.61 ± 1.81	30	70
3.	N95 (iii)	131.7 ± 24.12	33.31 ± 26.74	25	75
4.	NIOSH respirator	115.8 ± 19.43	34.63 ± 16.59	30	70

**Table 7:** Filtering efficiency of N95 FFRs against PM_2.5_.

S. N.	N95 FFRs	Without filtration (*μ*g/m^3^)	With filtration (*μ*g/m^3^)	TIL (%)	Efficiency (%)
1.	N95 (i)	49 ± 3.74	15.1 ± 2.15	31	69
2.	N95 (ii)	5.62 ± 0.78	1.8 ± 0.7	32	68
3.	N95 (iii)	138.1 ± 22	36.75 ± 20.43	27	73
4.	NIOSH respirator	122.1 ± 20.85	38.41 ± 14.59	31	69

**Table 8:** Filtering efficiency of PTCMs against PM_10_.

S. N.	Cloth masks (PTCMs)	Without filtration (*μ*g/m^3^) mean ± S.D	With filtration (*μ*g/m^3^) mean ± S.D	TIL (%)	Efficiency (%)
1.	PTCM 1	49.98 ± 2.83	13.82 ± 3.35	28	72
2.	PTCM 2	40.13 ± 3.01	13.56 ± 1.43	34	66
3.	PTCM 3	46.98 ± 1.84	15.73 ± 2.74	33	67
4.	PTCM 4	42.83 ± 2.32	17.71 ± 2.62	41	59
5.	PTCM 5	54.48 ± 8.04	20.84 ± 9.05	38	62

**Table 9:** Filtering efficiency of PTCMs against PM_2.5_.

S. N.	Cloth masks (PTCMs)	Without filtration (*μ*g/m^3^) mean ± S.D	With filtration (*μ*g/m^3^) mean ± S.D	TIL (%)	Efficiency (%)
1.	PTCM 1	41.64 ± 2.1	13.49 ± 3.34	32	68
2.	PTCM 2	34.72 ± 1.59	13.1 ± 1.31	38	62
3.	PTCM 3	57.38 ± 2.73	21.7 ± 2.59	38	62
4.	PTCM 4	36.31 ± 1.62	17.01 ± 2.07	47	53
5.	PTCM 5	45.31 ± 6.26	19.61 ± 7.86	43	57

**Table 10:** Correlation matrix showing a relationship between variables.

	Efficiency (PM_10_)	Efficiency (PM_2.5_)	Layers
Efficiency (PM_10_)	1		
Efficiency (PM_2.5)_	0.99^*∗*^	1	
Layers	0.92^*∗*^	0.94^*∗*^	1

## Data Availability

The data used to support the findings of this study are available from the corresponding author upon request.

## References

[1] Parajuly K. (2016). Clean up the air in Kathmandu. *Nature*.

[2] Regmi R. P., Kitada T., Kurata G. (2003). Numerical simulation of late wintertime local flows in Kathmandu valley, Nepal: implication for air pollution transport. *Journal of Applied Meteorology*.

[3] Kim K.-H., Kabir E., Kabir S. (2015). A review on the human health impact of airborne particulate matter. *Environment International*.

[4] Bajracharya I., Bhattarai N. (2016). Road transportation energy demand and environmental emission: a case of Kathmandu valley. *Hydro Nepal: Journal of Water, Energy and Environment*.

[5] Neupane B. B., Mainali S., Sharma A., Giri B. (2019). Optical microscopic study of surface morphology and filtering efficiency of face masks. *PeerJ*.

[6] Pacitto A., Amato F., Salmatonidis A. (2019). Effectiveness of commercial face masks to reduce personal PM exposure. *Science of the Total Environment*.

[7] Neupane P. R., Bajracharya I., Manandhar B. R., Prajapati M., Sujakhu H., Awal P. (2020). Estimating emission load from road transportation within the bhaktapur municipality, Nepal. *Journal of Environmental and Public Health*.

[8] Davidson C. I., Phalen R. F., Solomon P. A. (2005). Airborne particulate matter and human health: a review. *Aerosol Science and Technology*.

[9] Rajagopalan S., Al-Kindi S. G., Brook R. D. (2018). Air pollution and cardiovascular disease. *Journal of the American College of Cardiology*.

[10] Hadley M. B., Vedanthan R., Fuster V. (2018). Air pollution and cardiovascular disease: a window of opportunity. *Nature Reviews Cardiology*.

[11] Brook R. D., Newby D. E., Rajagopalan S. (2017). The global threat of outdoor ambient air pollution to cardiovascular health. *JAMA Cardiol*.

[12] Burnett R., Chen H., Szyszkowicz M. (2018). Global estimates of mortality associated with long-term exposure to outdoor fine particulate matter. *Proceedings of the National Academy of Sciences*.

[13] Lelieveld J., Evans J. S., Fnais M., Giannadaki D., Pozzer A. (2015). The contribution of outdoor air pollution sources to premature mortality on a global scale. *Nature*.

[14] Yang A., Cai L., Zhang R. (2017). Thermal management in nanofiber-based face mask. *Nano Letters*.

[15] Who (2018). Ambient (outdoor) air pollution. https://www.who.int/news-room/fact-sheets/detail/ambient-(outdoor)-air-quality-and-health.

[16] Shindell D., Kuylenstierna J. C. I., Vignati E. (2012). Simultaneously mitigating near-term climate change and improving human health and food security. *Science*.

[17] Tcharkhtchi A., Abbasnezhad N., Zarbini Seydani M., Zirak N., Farzaneh S., Shirinbayan M. (2021). An overview of filtration efficiency through the masks: mechanisms of the aerosols penetration. *Bioactive Materials*.

[18] Laumbach R., Meng Q., Kipen H. (2015). What can individuals do to reduce personal health risks from air pollution?. *Journal of Thoracic Disease*.

[19] Yang P., Seale H., Raina MacIntyre C. (2011). Mask-wearing and respiratory infection in healthcare workers in Beijing, China. *Brazilian Journal of Infectious Diseases*.

[20] Jamieson D. J., Honein M. A., Rasmussen S. A. (2009). H1N1 2009 influenza virus infection during pregnancy in the USA 2009 influenza virus infection during pregnancy in the USA. *The Lancet*.

[21] Webster R. G., Peiris M., Chen H., Guan Y. (2006). H5N1 outbreaks and enzootic influenza. *Emerging Infectious Diseases*.

[22] Murray M. J. (2015). Ebola virus disease. *Anesthesia & Analgesia*.

[23] Assiri A., Al-Tawfiq J. A., Al-Rabeeah A. A. (2013). Epidemiological, demographic, and clinical characteristics of 47 cases of Middle East respiratory syndrome coronavirus disease from Saudi Arabia: a descriptive study. *The Lancet Infectious Diseases*.

[24] Who (2019). *Coronavirus Disease 2019 (COVID-19): Situation Report*.

[25] Chen H., Guo J., Wang C. (2020). Clinical characteristics and intrauterine vertical transmission potential of COVID-19 infection in nine pregnant women: a retrospective review of medical records. *The Lancet*.

[26] Verma S., Dhanak M., Frankenfield J. (2020). Visualizing droplet dispersal for face shields and masks with exhalation valves. *Physics of Fluids*.

[27] Murray O. M., Bisset J. M., Gilligan P. J., Hannan M. M., Murray J. G. (2020). Respirators and surgical facemasks for COVID-19: implications for MRI. *Clinical Radiology*.

[28] Morais F. G., Sakano V. K., Lima L. N. de (2021). Filtration efficiency of a large set of COVID-19 face masks commonly used in Brazil. *Aerosol Science and Technology*.

[29] Phan T. L., Ching C. T.-S. (2020). A reusable mask for coronavirus disease 2019 (COVID-19). *Archives of Medical Research*.

[30] Eikenberry S. E., Mancuso M., Iboi E. (2020). To mask or not to mask: modeling the potential for face mask use by the general public to curtail the COVID-19 pandemic. *Infectious Disease Modelling*.

[31] Wang W., Wu Q., Yang J. (2020). Global, regional, and national estimates of target population sizes for covid-19 vaccination: descriptive study. *BMJ*.

[32] Wu H. l., Huang J., Zhang C. J. P., He Z., Ming W.-K. (2020). Facemask shortage and the novel coronavirus disease (COVID-19) outbreak: reflections on public health measures. *EClinicalMedicine*.

[33] Plana D., Tian E., Cramer A. K. (2021). Assessing the filtration efficiency and regulatory status of N95s and nontraditional filtering face-piece respirators available during the COVID-19 pandemic. *BMC Infectious Diseases*.

[34] Forouzandeh P., O’Dowd K., Pillai S. C. (2021). Face masks and respirators in the fight against the COVID-19 pandemic: an overview of the standards and testing methods. *Safety Science*.

[35] Kool J. L. (2005). Risk of person‐to‐person transmission of pneumonic plague. *Clinical Infectious Diseases*.

[36] Capps J. A. (1918). Measures for the prevention and control of respiratory infections in military camps. *JAMA, the Journal of the American Medical Association*.

[37] Dato V. M., Hostler D., Hahn M. E. (2006). Simple respiratory mask. *Emerging Infectious Diseases*.

[38] Beesoon S., Behary N., Perwuelz A. (2020). Universal masking during COVID-19 pandemic: can textile engineering help public health? Narrative review of the evidence. *Preventive Medicine*.

[39] Leung C. C., Lam T. H., Cheng K. K. (2020). Mass masking in the COVID-19 epidemic: people need guidance. *The Lancet*.

[40] Wang J., Du G. (2020). COVID-19 may transmit through aerosol. *Irish Journal of Medical Science*.

[41] Yan J., Guha S., Hariharan P., Myers M. (2019). Modeling the effectiveness of respiratory protective devices in reducing influenza outbreak. *Risk Analysis*.

[42] Konda A., Prakash A., Moss G. A., Schmoldt M., Grant G. D., Guha S. (2020). Aerosol filtration efficiency of common fabrics used in respiratory cloth masks. *ACS Nano*.

[43] Shakya K. M., Noyes A., Kallin R., Peltier R. E. (2017). Evaluating the efficacy of cloth facemasks in reducing particulate matter exposure. *Journal of Exposure Science and Environmental Epidemiology*.

[44] Chughtai A. A., Seale H., MacIntyre C. R. (2013). Use of cloth masks in the practice of infection control – evidence and policy gaps. *Int J Infect Control*.

[45] MacIntyre C. R., Seale H., Dung T. C. (2015). A cluster randomised trial of cloth masks compared with medical masks in healthcare workers. *BMJ Open*.

[46] Faridi S., Nodehi R. N., Sadeghian S. (2020). Can respirator face masks in a developing country reduce exposure to ambient particulate matter?. *Journal of Exposure Science and Environmental Epidemiology*.

[47] Yim W., Cheng D., Patel S. H., Kou R., Meng Y. S., Jokerst J. V. (2020). KN95 and N95 respirators retain filtration efficiency despite a loss of dipole charge during decontamination. *ACS Applied Materials & Interfaces*.

[48] Cherrie J. W., Apsley A., Cowie H. (2018). Effectiveness of face masks used to protect Beijing residents against particulate air pollution. *Occupational and Environmental Medicine*.

[49] Mueller W., Horwell C. J., Apsley A. (2018). The effectiveness of respiratory protection worn by communities to protect from volcanic ash inhalation. Part I: filtration efficiency tests. *International Journal of Hygiene and Environmental Health*.

[50] He X., Grinshpun S. A., Reponen T., McKay R., Bergman M. S., Zhuang Z. (2014). Effects of breathing frequency and flow rate on the total inward leakage of an elastomeric half-mask donned on an advanced manikin headform. *Annals of Occupational Hygiene*.

[51] He X., Reponen T., McKay R., Grinshpun S. A. (2014). How does breathing frequency affect the performance of an N95 filtering facepiece respirator and a surgical mask against surrogates of viral particles?. *Journal of Occupational and Environmental Hygiene*.

[52] Serfozo N., Ondráček J., Otáhal P., Lazaridis M., Ždímal V. (2017). Manikin-based size-resolved penetrations of CE-marked filtering facepiece respirators. *Journal of Occupational and Environmental Hygiene*.

[53] Cho K. J., Reponen T., McKay R. (2010). Large particle penetration through N95 respirator filters and facepiece leaks with cyclic flow. *Annals of Occupational Hygiene*.

[54] Balazy A., Toivola M., Reponen T., Podgórski A., Zimmer A., Grinshpun S. A. (2006). Manikin-based performance evaluation of N95 filtering-facepiece respirators challenged with nanoparticles. *Annals of Occupational Hygiene*.

[55] Rengasamy S., Eimer B. C., Szalajda J. (2014). A quantitative assessment of the total inward leakage of NaCl aerosol representing submicron-size bioaerosol through N95 filtering facepiece respirators and surgical masks. *Journal of Occupational and Environmental Hygiene*.

[56] Rengasamy S., Eimer B., Shaffer R. E. (2010). Simple respiratory protection - evaluation of the filtration performance of cloth masks and common fabric materials against 20-1000 nm size particles. *Annals of Occupational Hygiene*.

[57] Rogak S. N., Sipkens T. A., Guan M., Nikookar H., Vargas Figueroa D., Wang J. (2021). Properties of materials considered for improvised masks. *Aerosol Science and Technology*.

[58] Zhao M., Liao L., Xiao W. (2020). Household materials selection for homemade cloth face coverings and their filtration efficiency enhancement with triboelectric charging. *Nano Letters*.

[59] Bagheri M. H., Khalaji I., Azizi A. (2021). Filtration efficiency, breathability, and reusability of improvised materials for face masks. *Aerosol Science and Technology*.

[60] Gardner P. D., Eshbaugh J. P., Harpest S. D., Richardson A. W., Hofacre K. C. (2013). Viable viral efficiency of N95 and P100 respirator filters at constant and cyclic flow. *Journal of Occupational and Environmental Hygiene*.

[61] Clapp P. W., Sickbert-Bennett E. E., Samet J. M. (2021). Evaluation of cloth masks and modified procedure masks as personal protective equipment for the public during the COVID-19 pandemic. *JAMA Internal Medicine*.

[62] Ullah S., Ullah A., Lee J. (2020). Reusability comparison of melt-blown vs. nanofiber face mask filters for use in the coronavirus pandemic. *ACS Applied Nano Materials*.

[63] Duncan S., Bodurtha P., Naqvi S. (2021). The protective performance of reusable cloth face masks, disposable procedure masks, KN95 masks and N95 respirators: filtration and total inward leakage. *PLoS One*.

[64] Grinshpun S. A., Haruta H., Eninger R. M., Reponen T., McKay R. T., Lee S. A. (2009). Performance of an N95 filtering facepiece particulate respirator and a surgical mask during human breathing: two pathways for particle penetration. *Journal of Occupational and Environmental Hygiene*.

[65] Nallathambi G., S E., R K., D N. (2019). Multilayer nonwoven fabrics for filtration of micron and submicron particles. *Journal of Textile Engineering & Fashion Technology*.

[66] O’Kelly E., Pirog S., Ward J., Clarkson P. J. (2020). Ability of fabric face mask materials to filter ultrafine particles at coughing velocity. *BMJ Open*.

[67] Drewnick F., Pikmann J., Fachinger F., Moormann L., Sprang F., Borrmann S. (2021). Aerosol filtration efficiency of household materials for homemade face masks: influence of material properties, particle size, particle electrical charge, face velocity, and leaks. *Aerosol Science and Technology*.

[68] Zangmeister C. D., Radney J. G., Vicenzi E. P., Weaver J. L. (2020). Filtration efficiencies of nanoscale Aerosol by cloth mask materials used to slow the spread of SARS-CoV-2. *ACS Nano*.

[69] Kim M. C., Bae S., Kim J. Y. (2020). Effectiveness of surgical, KF94, and N95 respirator masks in blocking SARS-CoV-2: a controlled comparison in 7 patients. *Infectious Diseases*.

[70] Aragaw T. A. (2020). Surgical face masks as a potential source for microplastic pollution in the COVID-19 scenario. *Marine Pollution Bulletin*.

[71] Selvaranjan K., Navaratnam S., Rajeev P., Ravintherakumaran N. (2021). Environmental challenges induced by extensive use of face masks during COVID-19: a review and potential solutions. *Environmental Challenges*.

[72] Schnurr R. E. J., Alboiu V., Chaudhary M. (2018). Reducing marine pollution from single-use plastics (SUPs): a review. *Marine Pollution Bulletin*.

[73] Drabek J., Zatloukal M. (2019). Meltblown technology for production of polymeric microfibers/nanofibers: a review. *Physics of Fluids*.

[74] Dutton K. C. (2009). Overview and analysis of the meltblown process and parameters. *Analysis*.

[75] Fadare O. O., Okoffo E. D. (2020). Covid-19 face masks: a potential source of microplastic fibers in the environment. *Science of the Total Environment*.

[76] Min K., Weng X., Long P., Ma M., Chen B., Yao S. (2021). Rapid in-situ analysis of phthalates in face masks by desorption corona beam ionization tandem mass spectrometry. *Talanta*.

[77] Cole M., Webb H., Lindeque P. K., Fileman E. S., Halsband C., Galloway T. S. (2014). Isolation of microplastics in biota-rich seawater samples and marine organisms. *Scientific Reports*.

